# Cardioprotective Action of Glycyrrhizin on Diabetic Rats with Myocardial Remodeling

**DOI:** 10.1155/2021/6343677

**Published:** 2021-08-31

**Authors:** Fuxu Chen, Jie Song

**Affiliations:** ^1^Department of Cardiology, The Fourth Affiliated Hospital, Zhejiang University School of Medicine, N1 Shangcheng Road, Yiwu, Zhejiang, China; ^2^Electroencephalogram Room, The Fourth Affiliated Hospital, Zhejiang University School of Medicine, N1 Shangcheng Road, Yiwu, Zhejiang, China

## Abstract

**Introduction:**

Cardiovascular disorders are one of the prominent causes of risks of mortality which accounts for high rate of the deaths at a global level. The risk of deadly myocardial infraction grows because of diabetes which even causes the development of heart failure.

**Objective:**

The objective of this study was to understand and study the effect of glycyrrhizin on diabetes suffering rats with myocardial remodeling.

**Materials and Methods:**

Streptozotocin was used for induction of diabetes, and 8–12 weeks later, the assessment of inflammation, fibrosis, and cardiac damage was evaluated. Histopathological analysis and immunohistochemistry was performed to analyze the effect in various groups. Western blotting was performed to understand the proteins expressed in diabetes, and also, their expression was noted in treatment groups.

**Results:**

There was a significant rise in TNF-*α*, dense fibrosis, and collagen deposits in the STZ diabetes group. The effects of hyperglycemia were significantly improved in the glycyrrhizin-treated group. DAPI, BrDu, and caspase staining was also performed to understand apoptosis in tissues where the diabetic groups reported significant apoptosis, while the effects were significantly lower in the treated group.

**Conclusion:**

All the observations indicate that glycyrrhizin has cardioprotective action in diabetic rats with myocardial remodeling and is due to the inhibition of the NF-*κ*B signaling pathway in the myocardial layer.

## 1. Introduction

Approximately 30% of all deaths worldwide occur due to the cardiovascular disorders [1]. Acute myocardial infraction (AMI) is considered among those with the high mortality rate, and the infarct size is a chief determinant of prognosis in the patients. Restoration of the coronary blood circulation by the percutaneous coronary interventions (PCI) is considered to be the only clinically accepted and approved procedure to bound the infarct size [2]. The circulation of the high level of glucose might guide to the modified cardiomyocyte signaling which results in oxidative stress, fibrosis, and finally to the death of the myocyte cell [3].

The cardiac cells might face early transitions due to hyperglycemic conditions which may cause the discharge of important inflammatory mediators such as cytokines and chemokines [4]. The myocardial revascularization involvement is regularly demonstrating throughout the period of medication of patients with the persistent coronary artery disease (CAD). Advancement of angina and exercise potential in the patients with bounded symptoms is the most important observed advantages with these mediations [5].

The acute myocardial infarction heads to the ischemic necrosis of the myocardium which is considered to be harmful to the health of the mass population [6]. The timely widening of the coronary arteries in the patients suffering from the myocardial infraction diminishes the region of myocardial infraction, and there is an outstanding reduction in the mortality rate [7]. There is multiple known as well as unknown components that might affect the myocardial impairments followed by interferences.

However, this is still considered debatable as the diabetes mellitus might alter the myocardial responsibilities and possibly make the myocardium more prone to ischemic impairment [8, 9]. The cardiac muscles might even die, and the region of the myocardial necrosis leads to affect the prognosis of the patient suffering from myocardial infraction. In clinical practices, the myocardial damages lead to the disorder of the electric roles within the myocardial and cardiac deficiency along with arrhythmia. One of the crucial elements of root extraction from the liquorice is the acid, i.e., glycyrrhizin which is soluble in water. It consists of the glucuronic acid as well as the glycyrrhetinic acid [10].

The research study conducted by [11] demonstrates that the glycyrrhizin is a successful element in the liquorice that comprises of antiallergic, antioxidant, immunomodulatory, anticancer, antiulcer, and antiviral properties. The risk of lethal myocardial infarction and evolution of heart failure is intensified because of diabetes [12, 13]. The fundamental diabetic cardiomyopathy which is aggravated by other components such as the hypertension as well as ischemic heart disorders justifies the defective prognosis after the myocardial infarction.

The reactive oxygen species (ROS) as well as the reactive nitrogen species (RNS) is built as an outcome of hyperglycemia. This in turn persuades the p53 and the cytochrome-c moderated caspase-3-dependent apoptosis [14, 15]. Correspondingly, termination of myocardial cells in diabetes is averted by the utilization of the antioxidants and the caspase inhibitors which shows a spontaneous task for the apoptosis in the pathogenesis of diabetes-instigated cardiomyocyte loss.

## 2. Materials and Methods

Male Wistar rats weighing around 200–250 gm were obtained from the animal house. The rats were kept at a constant temperature of 25°C ± 2°C in cages. Food pellet and water were provided freely ad libitum, and 12 h light/12 h dark cycle was maintained. All experiments were duly approved by the ethical committee, and protocols were followed in accordance to National Institutes of Health Guidelines.

### 2.1. Induction of Diabetes

Type 2 diabetes was induced using streptozotocin 45 mg/kg via i.p., route. After 4 days of dose administration, the blood glucose levels were tested to ensure the induction diabetes in rats. Evaluation of inflammation and cardiac damage was done 8–12 weeks postinduction of diabetes. Animals were housed in the animal facility. Diabetic rats were administered Formulab Diet 5008 Purina ad libitum throughout the experiment. Accucheck glucometer (UK) was used for measuring the blood glucose levels via the tail region once in seven days.

### 2.2. Western Blotting

Rats tissues from the heart were harvested from all 3 groups and then processed for Western blotting. The primary antibodies used were CX43, GAPDH, CXCR4, RAGE, and TGF-*β* (Cell Signaling, Danvers, MA, USA) ET-1, NaV1.5, phospho-p38, Nrf2 (Thermo Fischer Scientific), and secondary antibodies used were anti-mouse IgG or anti-rabbit IgG (1 : 5000; Sigma Aldrich) and were used as control where the data's were compared with *β*-actin levels using the analytical software for processing images and determining the intensity and percentage of control.

### 2.3. Morphometric Analysis

At the end of experimentation, the rats were sacrificed, and tissues from the heart were fixed in 10% formalin solution. The tissues were embedded in paraffin, and 4 mm thick sections were cut. Myocyte obtained from sections were stained with hematoxylin and eosin, and captured images were analyzed.

Collagen fibers were stained and were quantified so as to measure the fibrosis. The collagen positive area was measured for all groups. Myocardial tissues were frozen and stained in oil-red and then washed and counterstained with hematoxylin. Images were captured using a microscope (Leica microsystems).

### 2.4. Immunofluorescence Staining

The paraffin sections were cut from control and treatment groups which underwent immunohistochemistry tests by using antigen retrieval methods. Tissue sections were incubated with primary antibodies for interleukin 6 (IL-6) (Genescript), interleukin 6 (IL-6) (Thermo Fischer), rabbit polyclonal collagens I and III (Thermo Fischer), and tumor necrosis factor TNF-*α* (Sino Biological) overnight, and then, they were stained with secondary antibodies at 370°C for thirty minutes. The stained sections were developed using diaminobenzidine and hematoxylin was used for counterstaining. All sections were viewed and captured using the ZEISS LSM 780 laser scanning microscope (Zeiss).

Sections were also stained with DAPI after three washings and then mounted on Fluoromount-G (Southern Biotech). Sections from cardiac tissue which were stained with troponin-I initially were analyzed for troponin intensity changes and compared with control, diabetic only, and diabetic rats with treatment for identification of the effects of glycyrrhizin on troponin-I in ventricular cardiac muscle.

Myocardial apoptosis: the effect of glycyrrhizin on apoptosis in cardiomyocytes in the diabetic rats was evaluated using DAPI, caspase, and BrDU staining.

### 2.5. Statistical Analysis

The results were expressed in mean ± SD. We used one-way ANOVA was used for checking the significant differences followed by the post hoc multiple comparison Tukey's test where *p* < 0.05 was considered as significant.

## 3. Results

The tissues collected from the ventricular heart in case of diabetic rats have shown a significant rise in collagen deposition which was improved in the glycyrrhizin treatment group (Figure 1). The collagen positive area was measured by positive trichrome staining. Means ± SE; *p* < 0.001; *n* = 6.

The expressions of TGF-*β* were increased in cardiomyocytes cells and cardiac tissues of the diabetic group which was improved with CXCR4 antagonist in case of the glycyrrhizin-treated group. TGF-*β*: fibrosis marker was evaluated in STZ-diabetic rats where a significant increase was shown on comparison to the control group. Treatment of four weeks in the glycyrrhizin-treated group caused a significant decrease in the TGF*β* expression in tissues of group II (treatment group) animals (Figures 2(a) and 2(b)).

Glycyrrhizin has shown increased levels in connexin43 (gap junction protein) in the cardiac tissues (Figure 3).

The stained cells in the diabetic group were higher on comparison to the normal control group, hence showing confirmed apoptosis in the myocardial region of the diabetic rats. Glycyrrhizin has shown a significant decrease in the apoptosis in myocardial cells, hence confirming the cardioprotective action of glycyrrhizin (Figure 4).

## 4. Discussion

Glycyrrhizin is a crucial water-soluble acid which is prominently used in Asian countries, in root extraction from liquorice. One of the major complicated disorders of chronic diabetes is myocardial fibrosis where many studies demonstrate high cardiac impairment postischemic results. Multiple clinical studies show the scenario of acute coronary syndromes which have direct impact over the high susceptibility of patients suffering from diabetes to a higher risk of heart failures.

The heart was isolated from rats and then fixed with formalin for further studies (Figures 5(a) and 5(b)). Deposition of collagen in cardiac fibrosis in the STZ diabetic rats, control group, and glycyrrhizin-treated groups was analyzed histopathologically, where it was found that collagen deposits were significantly higher in the diabetic groups as compared to the treated and control groups (Figure 6). Stained tissues were observed for fibrosis and collagen deposits.

The hyperglycemia condition mediates fibrosis in cardiac tissues which was analyzed by TGF-*β* (transforming growth factor beta), thus showing a significant increase in its expressions in the STZ rat cardiac tissues, while the expressions of TGF-*β* were significantly reduced in glycyrrhizin groups in treatment duration of four weeks. AC16 cardiomyocyte cells were also treated overnight with 25 mM of glucose and hyperglycemia cells were treated with AMD3100 (CXCR4 antagonist) to estimate the connection between TGF-*β* and CXCR4 pathways. Increase in TGF*β* expression was in hyperglycemic cardiomyocytes, while the treated group receiving AMD3100 had noted a decreased expression of TGF-*β* (Figure 2), hence showing the anti-inflammatory action of glycyrrhizin.

The regulation of cell adhesion for diabetic groups was performed by assessing the connexin43. Western blotting tests were performed for showing the reduced CX43 expression in heart tissues of diabetic rats on comparison to the control group. A restoration of the CX43 expression was shown in the treatment group. Western blot analysis was performed for tissue of STZ rats to understand the mechanisms involved in inflammatory responses during hyperglycemia and in cardiac fibrosis. A significant increase in expression of CXCR4 was found in diabetic groups versus the treated group, hence showing role of glycyrrhizin in CXCR4 expression, thus confirming the anti-inflammatory action of glycyrrhizin. Reduced CXCR4 expression showed the anti-inflammatory effect in diabetic rats with cardiac atrophy.

TGF*β* is a prime factor involved in contributing towards cardiac fibrosis. Hence, in this study, we concluded that STZ-induced hyperglycemia has shown activated cardiac fibroblasts and deposition of matrix proteins extracellularly. As the elevated factor TGF-*β* is responsible for fibrogenesis, the fibroblast production is seen to be prominent in diabetic rats but were ameliorated in the treatment group. Hence, we can say that there is an association of chemokines with cardiac fibrosis. Expressions of TGF-*β* in the myocardium were increased leading to fibrosis. Collagen fibers were also found significantly higher in the diabetic groups, whereas they were reduced in the glycyrrhizin group. Apoptosis was also noted in diabetic groups and was significantly reduced in the treated groups.

## 5. Conclusion

Hyperglycemia can lead to increased inflammation and oxidative stress which leads to cardiac remodeling and hence causes hypertrophy in the myocardium. The STZ rats showed an increased level of inflammation which may lead to cardiac injury and damage. The research concludes with findings about the anti-inflammatory and preventive cardiac damage properties of glycyrrhizin.

## Figures and Tables

**Figure 1:** Percentage of collagen positive area in all groups.

**Figure 2:** TGF-*β* expressions recorded by (a) Western blotting and (b) quantification in control, diabetic, and treated groups.

**Figure 3:** Glycyrrhizin alters CXCR4 expressions in myocardial tissues in STZ-diabetic rats.

**Figure 4:** Immunofluorescent staining of tissues from all groups with DAPI, caspase, and BrDU for analysis of apoptosis.

**Figure 5:** Isolated heart from the experimental rats. (a) Freshly isolated heart for fixing. (b) Fixed organ in 10% formalin solution.

**Figure 6:** Histological analysis of tissues in all groups with collagen and fibrosis assessment.

## Data Availability

The data used to support the results of the study are available from the first author or corresponding author upon request.

## Abbreviations

STZ: Streptozotocin
TGF-*β*: Transforming growth factor-beta
CXCR4: Chemokine receptor type 4
DAPI: 4′,6-Diamidino-2-phenylindole
BrDU: Bromodeoxyuridine.
